# Recognition of Fetal Facial Ultrasound Standard Plane Based on Texture Feature Fusion

**DOI:** 10.1155/2021/6656942

**Published:** 2021-06-03

**Authors:** Xiaoli Wang, Zhonghua Liu, Yongzhao Du, Yong Diao, Peizhong Liu, Guorong Lv, Haojun Zhang

**Affiliations:** ^1^College of Medicine, Huaqiao University, Quanzhou 362021, China; ^2^Department of Ultrasound, Quanzhou First Hospital Affiliated to Fujian Medical University, Quanzhou 362021, China; ^3^Collaborative Innovation Center for Maternal and Infant Health Service Application Technology, Quanzhou Medical College, Quanzhou 362021, China; ^4^College of Engineering, Huaqiao University, Quanzhou 362021, China; ^5^Department of Ultrasound, The Second Affiliated Hospital of Fujian Medical University, Quanzhou 362021, China; ^6^Biomedical Ultrasound Laboratory, The University of Southern California (USC), Los Angeles, USA

## Abstract

In the process of prenatal ultrasound diagnosis, accurate identification of fetal facial ultrasound standard plane (FFUSP) is essential for accurate facial deformity detection and disease screening, such as cleft lip and palate detection and Down syndrome screening check. However, the traditional method of obtaining standard planes is manual screening by doctors. Due to different levels of doctors, this method often leads to large errors in the results. Therefore, in this study, we propose a texture feature fusion method (LH-SVM) for automatic recognition and classification of FFUSP. First, extract image's texture features, including Local Binary Pattern (LBP) and Histogram of Oriented Gradient (HOG), then perform feature fusion, and finally adopt Support Vector Machine (SVM) for predictive classification. In our study, we used fetal facial ultrasound images from 20 to 24 weeks of gestation as experimental data for a total of 943 standard plane images (221 ocular axial planes, 298 median sagittal planes, 424 nasolabial coronal planes, and 350 nonstandard planes, OAP, MSP, NCP, N-SP). Based on this data set, we performed five-fold cross-validation. The final test results show that the accuracy rate of the proposed method for FFUSP classification is 94.67%, the average precision rate is 94.27%, the average recall rate is 93.88%, and the average *F*1 score is 94.08%. The experimental results indicate that the texture feature fusion method can effectively predict and classify FFUSP, which provides an essential basis for clinical research on the automatic detection method of FFUSP.

## 1. Introduction

Ultrasound has been used for prenatal observation, measurement, and diagnosis of fetal diseases for nearly 30 years due to its advantages of low cost, portability, no radiation, and real-time imaging capabilities. Historical experience and the majority of facts show that ultrasound diagnosis is very safe and effective [1–3]. Due to the large population base in our country, there are many abnormal births every year, causing numerous medical disputes and a heavy burden on the family and society, affecting the quality of the national population [4]. Prenatal diagnosis is the key to screening for fetal abnormalities. Parents-to-be can make reproductive decisions for their unborn children on a legal basis based on the screening results [5]. Therefore, taking effective measures to improve prenatal ultrasound diagnosis and reduce the missed diagnosis rate of fetal malformations is of great value in reducing newborn congenital disabilities.

The standard planes of fetal ultrasound play a decisive role in understanding fetal anatomy and tissue development [6, 7]. Since there is more amniotic fluid in pregnant women during the middle pregnancy period, the fetus is relatively mature, and some planes can be readily displayed. It is typical to use ultrasonic images of the fetus during the middle pregnancy period prenatal ultrasound diagnosis. The standard planes can be screened by doctors to effectively detect abnormal fetuses, and timely planning of treatment plan can improve the fetus' survival rate during the perinatal period, which is of great significance for eugenics [8]. However, in the prenatal diagnosis' clinical practice, a sonographer or radiologist obtains a two-dimensional image frame by manually positioning an ultrasound probe [8–10], which contains various types of standard ultrasound planes of the fetus as required. This manual method of obtaining the standard planes is time-consuming and highly dependent on the sonographer's skill and experience [11]. In this situation, it is crucial to study an objective and efficient method to recognize fetal ultrasonic standard planes automatically.

The FFUSP consists of three elemental planes (Figure 1): the ocular axial planes (OAP), the median sagittal planes (MSP), and the nasolabial coronal planes (NCP). Although the fetus' facial part develops late compared with the ordinary images, FFUSP is a good plane for observing the fetus' facial contour and screening various fetal cleft lips. Many labial and facial abnormalities are displayed in FFUSP. Therefore, ultrasonic physicians can evaluate the fetus' facial contour based on FFUSP images and screen and diagnose the facial structural abnormalities such as nose, lip, and eye by measuring the relevant parameters [8, 9]. The applicable specifications were formulated for the fetus' standard clinical planes, and the application [4, 12, 13] improved the prenatal diagnosis of fetal abnormalities and laid the foundation for the standardized training and quality control of prenatal screening for fetal anomalies. However, the traditional method of obtaining standard planes relies on the doctors' professional knowledge and clinical experience for a more subjective evaluation. As it cannot guarantee that the operators have the same level of energy and experience, this method often leads to large errors. Besides, the purely artificial evaluation method takes a large amount of time, which reduces clinical diagnosis efficiency [14].

Although the professional skills of obstetricians have been greatly improved with the popularity of prenatal ultrasound diagnosis and standardized training of ultrasound doctors in recent years, there are still some factors affecting the fetal ultrasound in the daily ultrasound work, such as the influence of the resolution of ultrasound equipment, the experience, concentration, energy, and sense of responsibility of the ultrasound doctors. This study is aimed at improving the recognition and classification efficiency of standard planes of fetal facial ultrasound and reducing the impact of human factors on the quality of fetal ultrasound. From the perspective of how to identify and obtain various types of standard ultrasonic planes of fetal facial, we should take measures to minimize the dependence of obtaining standard ultrasonic planes on ultrasonic doctors' qualifications and the influence of different ultrasonic devices to improve the efficiency of prenatal ultrasonic examination.

## 2. Related Works

In the prenatal ultrasound examination, many types of planes need to be used, and doctors usually acquire the standard fetal ultrasound planes manually. Because it is challenging to acquire the fetal ultrasound planes, and there are differences among different ultrasound doctors in clinical work experience, as well as different levels of cognition on the anatomical structure and characteristics of fetal planes, there are problems of small interclass differences and large intraclass differences among the obtained various planes [14, 15]. Manually obtaining the standard planes requires a large number of repetitive operations by doctors. Simultaneously, the examination time of pregnant women is too long for clinical efficiency to be improved. Therefore, studying the automatic recognition and classification of fetal ultrasound standard planes can effectively improve prenatal diagnosis efficiency and is of great significance for clinical prenatal ultrasound diagnosis.

With the application of artificial intelligence (AI) in various fields, AI has made outstanding achievements in medical image recognition and analysis in recent years. The primary research to realize AI and ultrasonic scanning mainly focus on the automatic or semiautomatic identification and classification methods of ultrasonic standard planes in different parts. The challenges are as follows: first, the imaging principle of ultrasonic images makes ultrasonic images have high noise and low contrast [16, 17]. Simultaneously, due to the noise or shadow caused by different operators, different scanning angles, and scales, the ultrasonic image features are difficult to distinguish [18]. Generally speaking, automatic recognition and standard plane classification methods can be divided into image recognition and classification methods based on traditional manual features and image recognition and classification methods based on depth features.

Image recognition and classification based on traditional manual features are mainly divided into three steps: feature extraction, feature coding, and feature classification [19–22]. In 2012, Liu et al. [23] fitted and located the standard plane of fetal head through activity expression model and used the Active Appearance Models (AAM) method to find the specific structure unique to the correct scanning plane. In 2013, Ni et al. [24] proposed the first automatic positioning scheme of the upper abdomen's standard plane, using the prior knowledge of clinical anatomy; the radial model was used to describe the positional relationship of critical anatomical structures in the abdominal plane, thus, realizing the standard plane positioning. In 2014, Lei et al. [25] proposed combining the underlying features and multilayer Fisher Vector (FV) feature coding to construct the full image features and assisted by an SVM classifier to locate the standard fetal plane. The limitation of this method is that the underlying features have certain limitations in feature representation, so the algorithm's performance still needs to be improved. In 2015, Lei et al. [26] proposed a new recognition method of fetal facial standard plane. The image features were extracted by densely sampled root scale-invariant feature transform (Root SIFT), then coded by FV, and classified by SVM. The final recognition accuracy is 93.27%, and the mean average precision (MAP) is 99.19%. In 2016, Liu et al. [27] put forward a three-dimensional ultrasound automatic calibration method of three orthogonal reference standard planes of the fetal facial. They designed the system, which realized the automatic calibration of three reference standard planes: median sagittal plane, denomination coronal plane, and horizontal transverse plane. In 2017, J. Alison Noble of Oxford University, UK [28] predicted the visibility, position, and direction of fetal heart ultrasound images by using the Return Woods method to determine the fetal heart's standard plane from each video frame and obtained the same accuracy as experts. In addition, there are some works related to our method. For example, in 2017, Fekri-Ershad and Tajeripour [29] proposed an improved LBP algorithm, which can not only extract color features and texture features jointly but also resist impulse noise effectively. Essentially, it is a breakthrough of the LBP algorithm. In 2020 [30], he further proposed a high-precision classification method of bark texture based on improved local ternary pattern (ILTP). This paper not only introduced some updated versions of LBP and LTP but also inspired our experiments.

After 2012, deep learning (DL) began to emerge, and automatic recognition and classification technology based on deep learning was gradually introduced into the task of automatic recognition and classification of the standard ultrasonic plane. The deep learning method is mainly divided into two steps: first, the image is trained by the depth network model, the depth features of the image are extracted, and then the trained depth network is used to identify or classify the image. In 2014, Chen et al. [31] proposed a migration learning framework based on a convolutional neural network (CNN), which used a sliding window classification to locate a cut plane. In 2015, Chen et al. [32] put forward a migration learning (ML) framework based on a cyclic neural network, which combined CNN with a long and short time series model to locate the OAP in fetal ultrasound video. In the same year, Ni Dong Research Group of Shenzhen University [33] located the fetal abdominal standard plane (FASP) of the fetus through a pretrained neural network, using two neural networks, in which T-CNN was used to extract ROI area and R-CNN was used to identify the standard plane. The results show that the accuracy of ROI extraction by T-CNN reaches 90%, and the recognition rate by R-CNN reaches 82%. In 2017, Chen et al. [34] proposed a composite neural network to automatically identify fetal ultrasound standard planes: fetal abdominal standard plane (FASP), fetal facial axial standard plane (FFASP), and fetal four-chamber view standard plane (FFVSP) from ultrasound video sequences. In the end, the recognition rate of the FASP standard plane reaches 90%, the FFASP recognition rate reaches 86%, and FFVSP recognition rate reaches 87%. In the same year, Baumgartner et al. [2] of Imperial College London proposed a neural network model called SonoNet for real-time detection and localization of fetal ultrasound standard scanning planes. This method can automatically detect the position of 13 kinds of standard fetal views in two-dimensional ultrasound data and locate the fetal structure through the boundary box; in the real-time detection of real classification experimental modeling, the average *F*1-score is 0.798, the accuracy rate is 90.09%, and the accuracy rate of localization task reaches 77.8%. In 2018, Yu et al. [35] proposed that the automatic recognition of fetal facial ultrasonic standard plane was based on the framework of deep convolution neural network (DCNN), and the recognition rate of the fetal facial standard plane was as high as 95% by using this method. Besides, in recent years, researches on the measurement of biological parameters [36–38] and the detection of vital anatomical structures [39, 40] of fetal ultrasound images have emerged one after another.

The above work has achieved good results in the corresponding research fields. Still, there are also one or more shortcomings, such as

- The research method is low in universality and not suitable for positioning other types of fetal standard planes
- The adopted method needs manual intervention and has a low automation level and limited clinical practical value
- Due to the model's defects, the accuracy of standard plane positioning is easily affected by accumulated errors
- The convolutional neural network model is challenging to train, complicated in-process, and slow in operation

Given the current research status of ultrasonic planes of fetal facial, and considering the characteristics of FFUSP, that is, the number of standard planes is small, and the characteristics of the three types of standard planes are quite different, we propose an ultrasonic standard plane recognition and classification method that is relatively simple in process, fast in operation speed, and suitable for other parts of the fetus. In this study, a method based on image texture feature fusion and Support Vector Machine was used to identify and classify the prenatal FFUSP. This proposed method was evaluated in terms of classification accuracy, precision, recall, and *F*1-score through experiments. The processing flow chart of the method in this study is shown in Figure 2.

## 3. Methods and Materials

### 3.1. Image Acquisition and Experimental Data Distribution

#### 3.1.1. Image Acquisition Process

This study was approved and audited by the Ethics Committee of School of Medicine, Huaqiao University, and all the relevant topics were notified of approval. The data of three types of standard ultrasound planes (OAP, MSP, and NCP) and the nonstandard plane (N-SP) of fetal facial involved in the experiment were provided by Three Grade A hospitals (Quanzhou First Hospital Affiliated to Fujian Medical University). With the pregnant women's permission under examination, the professional ultrasound doctors recorded and saved the ultrasound scanning video through Philips EPIQ5 ultrasound instrument and GE Volusen E8 ultrasound instrument and further screened the pictures in the scanning video to ensure the accuracy of the experimental data to the greatest extent.

#### 3.1.2. Image Inclusion and Exclusion Criteria

Image inclusion criteria:

- The image was clear, and the target structure located in the center of the image accounted for more than 1/2 of the whole image. The background was pure and free of artifacts
- No superimposed color flow image in the image, no measurement caliper, text identification, and other artificial comments
- Postpartum confirmed fetal without facial and other structural abnormalities

Image exclusion criteria:

- The images were blurred and smeared due to the obesity of pregnant women, image jitter, and other reasons. The target structure was not displayed
- Ultrasound or postpartum confirmed fetal abnormalities

#### 3.1.3. Experimental Data

Finally, 943 pieces of data from the three types of standard planes and 350 pieces of data from nonstandard planes of fetal facial ultrasound were added to the experiment. The data proportion distribution of the four types of planes and the number of data sets randomly divided by five-fold cross-validation are shown in Table 1. In the experiment, each data set was used as the test set in sequence, and the remaining four groups were used as the training set. The final experimental results were the average of the five experiments. The experimental set images were from the fetal images of 20–24 weeks of pregnancy examined in the Ultrasound Medical Imaging Workstation of the Department of Ultrasound Medicine of Quanzhou First Hospital from January 2019 to December 2019. Besides, all the personal information concerning the subjects in the pictures was deleted, thus, protecting the subjects' privacy.

#### 3.1.4. Characteristics and Clinical Significance of Fetal Facial Ultrasound

Figure 1 shows three types of standard planes of fetal facial: OAP, MSP, and NCP. We have marked the crucial structures on the images of the three types of standard planes. The OAP is the reference plane for the fetal facial, and such standard planes require that the crystalline lens (CL) and eyeball (EB) be approximately the same size in the same plane. Clinically, doctors can diagnose fetal eye deformity, congenital cataract, abnormal eye distance, and other diseases through the plane. MSP is an excellent plane to observe the fetal facial contour, requiring frontal bone (FB), nasal bone (NB), apex nasi (AN), and lower jawbone (LJ) to be visible on such standard planes, and requiring that the lower jawbone be hyperechoic at origin only and not show nostrils. Doctors can diagnose fetal frontal protrusion, cleft lip and palate, and other facial abnormalities through this type of plane. The NCP is a routine plane for screening various cleft lips. Such standard planes obtained are required to show the contour of the nose and lips, including the structure of the apex nasi (AN), nasal column (NC), nostrils (Nos), upper lip (UL), lower lip (LL), and the mandible (MD). Therefore, this plane can be used to screen cleft lip and screen other facial abnormalities such as nasal abnormalities and facial deformities.

As all experimental data in this study were obtained from the ultrasonic scanning video of fetal facial, the nonstandard planes shown in Figure 3 were mainly divided into two types: nonstandard planes similar to the standard plane morphology and the other being the nonstandard planes with other morphology. The N-SP similar to the standard plane morphology had a very similar structure to the standard plane, which significantly increased this experiment's difficulty. This study's focus was not only how to distinguish the three standard planes but also how to distinguish the standard plane from the N-SP with different forms.

### 3.2. Methods

This study is aimed at realizing the recognition and classification of the standard ultrasound planes of fetal facial based on the simple process and fast operation of the experimental method model. In this study, Local Binary Pattern (LBP) [41] and Histogram of Oriented Gradient (HOG) [42] were used to extract the texture features of the images, and the Support Vector Machine (SVM) [43] was used to learn the texture features. Finally, the recognition and classification of the ultrasonic plane of fetal facial were achieved. Further, we compared it with other mainstream classifiers through experiments. Below, we will introduce the method used in this research.

#### 3.2.1. Data Preprocessing

In the original ultrasound images, in addition to the speckle noise inherent in the ultrasound images and the differences between images caused by different instruments, the different sizes of images, the shooting angles of the images, and the scaling of vital anatomical structures can also interfere with the judgment of the standard plane. We cut out the target pictures from the original experimental pictures by customizing the edge detection in the collected original experimental pictures to solve this problem. The picture obtained in the step has the advantages: (1) subject information in the picture is eliminated; (2) the vital anatomical structure is more prominent. Further, given the speckle noise inherent in the image and the difference in the gray distribution of different pictures, we perform the gray normalization on the target picture, which effectively balances the image's gray distribution and minimizes the image distortion. After pretreatment, the picture's size finally added into the experiment was further reduced to 512∗512 pixels.

#### 3.2.2. Texture Feature Extraction

*(1) Local Binary Pattern (LBP) [41]*. The LBP [41] is an operator used to describe local texture features of the image, which has obvious advantages such as rotation invariance and gray invariance. The original local binary pattern operator is defined on a central pixel and its surrounding rectangular neighborhood system with 3 × 3 pixels. For each central pixel, each neighborhood pixel's values are compared with the gray value of the central pixel as a threshold value to form binary quantization. The pixel value larger than or equal to the central pixel is coded as 1, and the value smaller than the central pixel is coded as 0, thus, forming a local binary pattern. After the binary pattern is generated, serial coding is carried out in a counterclockwise direction with the 0 direction of the current center pixel as the starting point to obtain a binary number. The decimal number corresponding to the binary number is used to identify the current center pixel uniquely. After that, Ojala et al. [44] modified LBP and formed a systematic theory in order to improve the limitation that the original LBP could not extract the large-size structural texture features.

In our experiments, the specific calculation formula is as follows:

(1) $$\begin{array}{c} {\text{LBP}}_{P,R}\left(x_{c},y_{c}\right)=\overset{P-1}{\underset{i=0}{\sum }}s\left(g_{i}-g_{c}\right)2^{i},\\ s\left(g_{P}-g_{c}\right)=\left\{\begin{array}{c} 1,\left(g_{P}-g_{c}\right)\geq 0,\\ 0,\left(g_{P}-g_{c}\right)<0, \end{array}\right. \end{array}$$

Where *R* is the radius of the neighborhood circle, and *P* represents the number of neighbors around the central pixel (*x*_*c*_, *y*_*c*_). *g*_*c*_ is the gray value of the central pixel, and *g*_*i*_ represents the gray value of neighboring pixels. In our experiments, *R* = 1 and *P* = 8.

*(2) Histogram of Oriented Gradient (HOG) [42]*. HOG is a commonly used feature to describe the local texture of images in computer vision and pattern recognition, and its application results in face recognition and target tracking are remarkable. The feature descriptor calculates the values of gradients in different directions in a particular area of the picture and then accumulates them to obtain histograms, which represent this area as features.

For each central pixel, the idea of HOG is to convolute the image with gradient operators [−1 0 1] and [−1 0 1]_*T*_ to obtain the gradient amplitude *m*(*x*_*i*_) and gradient direction *θ*(*x*_*i*_) of any pixel *x*_*i*_. The specific calculation formula is as follows:

(2) $$\begin{array}{c} \left\{\begin{array}{c} I_{x}=F\left(x+1,y\right)-F\left(x-1,y\right),\\ I_{y}=F\left(x,y+1\right)-F\left(x,y-1\right), \end{array}\right.\\ m\left(x,y\right)=\sqrt{I_{x}^{2}+I_{y}^{2}},\\ \theta \left(\text{x},\text{y}\right)=\tan^{-1}{\frac{I_{y}}{I}}_{x}\in \left[0,\left.360^{{}^{\circ}}\right)\right.\text{ or }\left[0,\left.180^{{}^{\circ}}\right)\right.. \end{array}$$

In the phase of texture feature extraction, we divide the target image into *n* cells which size is a × a pixel, and then traversed each pixel point on the *n* cells to generate the corresponding feature matrix. The generated features are then reshaped into a number of adjacent cell arrays to access the histogram of each cell (as shown in Figure 4). Histogram parameters determine how to aggregate the distribution of binary patterns and directional gradient histograms on the image to generate output features. The binary pattern is calculated for each cell, and the direction gradient histogram is obtained. Each cell has the same size and does not overlap to obtain different position information. Calculate the number of cells as imageSize/CellSize.

#### 3.2.3. Texture Feature Fusion

In the texture feature extraction step, the cells of LBP and HOG are two-element vectors specified in pixel units. To capture large-scale spatial information, we can appropriately increase the cell size, but it may lose small-scale details while increasing the cell size. Therefore, we defined the LBP and HOG cell size (CellSize) in the experiment as [72,72] through parameter optimization. Due to the diversity of images, the normalization of feature vectors can effectively remove background information and improve the image recognition rate. At the same time, normalization makes the feature vectors between different dimensions have a certain numerical comparison, which greatly improves the accuracy of classification. This step is a routine step in the process of extracting texture features. Performing L2 normalization on the histogram corresponding to each cell unit, and reshaping the LBP feature vector and the HOG feature vector obtained from each picture to form 1 × *N* and 1 × *M* feature vectors, wherein *N* and *M*, respectively, represent the number of LBP features and the number of HOG features. Finally, the LBP features and HOG features are fused into a feature vector of 1 × (*N* + *M*) as the input classifier's texture feature vector.

#### 3.2.4. Multiclassification Classifier

The Support Vector Machine's (SVM) [43] main task is to correctly separate data sets. The idea is to find a super plane between classes in *n*-dimensional space to correctly separate positive and negative samples, which is the SVM classifier. The SVM classifier we found is used to solve the problem of binary classification. For the four classes involved in this research, we design a binary classifier between every two classes. Classifier 1: *A* as a positive set, and *B*, *C*, *D* as a negative set; classifier 2: *B* as a positive set, and *A*, *C*, *D* as negative set; classifier 3: *C* as a positive set, and *A*, *B*, *D* as negative set; classifier 4: *D* is taken as a positive set, and *A*, *B*, *C* are taken as a negative set. Finally, the four subclassifiers were combined to form a multiclass classifier for automatic recognition and classification of the standard ultrasonic plane of the fetal facial. When classifying an unknown sample, the sample is taken into a first classifier 1. Suppose the classifier determines that the sample is a positive set. In that case, the sample is output as *A*. If the sample is determined as a negative set, the sample is continuously taken into classifier 2, and so on, until the classifier *n* gives a classification label of the sample, and the final classification result is output.

## 4. Experiments and Results

### 4.1. Experimental Environment

The specific hardware configuration of the computer equipment used in this experiment is as follows: Intel(R) Core (TM) i7-7700 is used for CPU, NVIDIA GeForce GTX-1080Ti is used for GPU, and the video memory is 11G and the memory is 32 G. The computer's operating system is 64-bit Windows 10, and the programming software is MATLAB R2018b.

### 4.2. Evaluation Index

This paper evaluates the model by calculating the precision, recall, *F*1-score, and accuracy of the prediction labels. *F*1-score is one of the commonly used comprehensive evaluation indexes (F-Measure), which is the weighted harmonic average of recall and precision, to prevent the contradiction between recall and precision from objectively evaluating the performance of the model. A higher value of *F* proves that the model is more effective. The relevant formula is defined as follows:

(3) $$\begin{array}{c} \text{Precision}=\frac{\text{TP}}{\text{TP}+\text{FP}},\\ \text{Recall}=\frac{\text{TP}}{\text{TP}+\text{FN}},\\ F1-\text{score}=\frac{2\times \text{Precision}\times \text{Recall}}{\text{Precision}+\text{Recall}},\\ \text{Accuracy}=\frac{\text{TP}+\text{TN}}{\text{TP}+\text{FN}+\text{FP}+\text{TN}}. \end{array}$$

In the formula, TP means the number of positive cases predicted as positive cases, FP means the number of negative cases predicted as positive cases, TN means the number of positive cases predicted as negative cases, and FN means the number of negative cases predicted as negative cases.

### 4.3. Experimental Results

Through the experimental process in Figure 2, we conducted the experiments on four classes of planes. The experimental results are shown in Table 2, where Group represents the experimental group in the five-fold cross-validation and precision, recall, and *F*1-score, respectively, represent the average values of the four classes of planes in each group on the corresponding indicators. Using this study's method, the overall recognition accuracy of the ultrasonic plane of the fetal facial reaches 94.67%. It could be clearly seen that each group performed well in all evaluation indexes, and all indexes were above 91.00%. Group A and group E performed well, followed by the other three groups. Finally, the five-fold cross-validation experiment's average results were more than 93.00%, indicating that the experimental method performed better.

#### 4.3.1. Comparative Experiments

To further illustrate the advantages of choosing the fusion of LBP [41] and HOG [42], we separately conducted experiments on the LBP feature [41] and HOG feature [42] under the same experimental environment and dataset settings and obtained the experimental results.  Table 3 shows the results of the single feature comparison experiment.

It can be seen from Table 3 that the LBP feature [41] and HOG feature [42] alone also achieve good results, especially when the LBP feature [41] is used alone, the precision, recall, and *F*1-score of each group are more than 90.00%. The overall accuracy is very close to the results in Table 2. However, the average precision, recall, *F*1-score, and accuracy of the five-fold cross-validation are lower than this experimental method's results. Moreover, when using the HOG feature alone [42], all aspects of the performance are significantly worse than the texture feature fusion method. Notably, when using other classifiers, the performance of the texture feature fusion method is superior to individual features. Combined with Table 2, we can conclude that the texture feature fusion method in this study is superior to the single texture feature method. The LBP feature [41] and HOG feature fusion [42] perform best in recognizing standard planes of fetal facial.

After the effect of a single texture feature on the experimental results is verified, we further explore the effect of different classifiers on the experiment's efficiency. In this stage, we introduce the *K*-nearest neighbor classifier (KNN) [45] and naive Bayes classifier (NB) [46]. For the introduced classifier, we also find the optimal cell size of the texture feature corresponding to it by parameter optimization, where the optimal cell size of the texture feature corresponding to the KNN classifier is [56,56] pixels, and the optimal cell size of the texture feature corresponding to the NB classifier is [40] pixels. On this basis, different classifiers are compared with different texture features one by one in the experiment. The experimental results show the accuracy, recall, *F*1-score, and accuracy are shown in Table 3.

The data shown in Table 3 shows that the KNN classifier [45] performs well in the classification experiment of the ultrasonic plane of fetal facial, and all the indicators are stable at about 88%; The NB classifier [46] performed generally, and the SVM classifier [43] performed best. Besides, in terms of the time consumption of this experiment, SVM < NB < KNN. The above results have fully demonstrated the necessity of applying the SVM classifier to the FFUSP classification.

In our experiment, the number of neighbors corresponding to LBP_*P*,*R*_ was *P* = 8, and the radius was *R* = 1. To demonstrate the superiority of this parameter in the experiment of the fetal facial ultrasonic plane, we obtained the LBP performance in different (*P*, *R*) values through a comparative experiment. The results of this experimental method in different (*P*, *R*) values are shown in Table 4.

Looking at Table 4, it is not difficult to find that when *P* = 8 (or 16) and *R* = 1 (or 2), the experimental classification accuracy all above 94.00%, and when *P* and *R* are larger (e.g., *P* = 24 and *R* = 3), the four indexes corresponding to the experimental results all decrease. Besides, when the values of *P* and *R* are larger, the stability of cross-validation results is improved, but the experimental processing will be more time-consuming. The LBP with different (*P*, *R*) values is superimposed, and each combination method has achieved good experimental results. The reasons may lie in: on the one hand, the sensitivity of LBP to (*P*, *R*) values in this experiment is small; on the other hand, the experimental data set is not large enough, which may not objectively reflect the influence of different (*P*, *R*) values.

#### 4.3.2. Parameter Optimization and Stability Test

In the texture feature extraction stage, we need to divide the target image into cells to access the histograms on each cell, and the size of the cell will directly affect the formation of feature vectors, thus, affecting the image recognition and classification results. In the experimental data shown in this paper (Table 2), the cell size is set to [72,72] pixels. To find this optimal parameter, we defined the cell size as the range of [20,20]-[100,100]. A total of 41 × 5 experiments were conducted with [20] pixels as the starting point, [100,100] pixels as the endpoint, and [2] pixels as the difference value. Finally, the classification experiment performed best when the cell size was [72,72].

If the cell size is changed, will the experimental results show serious deviation and directly indicate that the model's performance is not excellent? To verify this problem's existence, we compared the experimental results corresponding to each group of parameters in the parameter optimization process. The average accuracy of the five-fold cross-validation experiment under 41 groups of parameters is in the range of 92.73%-94.67%. The average precision is in the range of 92.25%-94.34%, the average recall is in the range of 91.65%-93.87%, and the average *F*1-score is in the range of 91.84%-94.03%. In Figure 5, with the pixel size of [72,72] as the center, we visually compare the experimental results corresponding to 12 groups of parameters (with one side at an interval of two pixels) on the left and right sides, respectively.

We can conclude that the setting of cell unit size affects the experimental results to a certain extent. Still, it is not the most crucial factor that affects the classification effect of the FFUSP using texture features in this study. The method used in this study has a certain stability.

### 4.4. Discussion and Future Work

Prenatal ultrasound is one of the essential means to screen for fetal abnormalities. Clinically, doctors have found that 32–39 classes of planes of the fetus [8, 9] are significant in the ultrasonic examination of the fetus, and most structural malformations of the fetus can be screened and diagnosed through these planes. Specifically, the fetal facial is an acceptable plane for observing the fetus' facial contour and screening various fetal cleft lips. Many labial and facial abnormalities are displayed on the fetal face. However, currently, doctors who acquire FFUSP by traditional methods cannot adapt to rapid and efficient ultrasonic examination, so it is crucial to find an automatic and rapid FFUSP recognition method. We have found a method model suitable for solving the problem of automatically identifying and obtaining the three standard planes of the fetal facial.

The experimental results show that the traditional method of texture feature fusion with mainstream classifier can effectively and automatically identify and classify FFUSP images. In particular, for the recognition and classification problems involving fewer categories, the traditional texture features largely overcome the difficulties in training the convolutional neural network model, the complexity of the process, the slow operation, and other problems. In this paper, the fusion of LBP and HOG and the adoption of SVM recognition and classification have achieved excellent results.

In the process of predicting and classifying the ultrasonic planes of fetal facial by this research method, we performed index transformation *y*_*i*_ = *e*^*x*_*i*_^ of the prediction values *x*_*i*_(*i* = 1, 2, 3, 4) given by the classifier to obtain the similarity (0 ~ 1) of the images to be classified and the four types of images, respectively. The last classification label of the pictures to be classified corresponds to the final decision with the highest similarity, and the classification result is obtained. The prediction classification process is shown in Figure 6. The significance of converting the predicted values into similarity is not only to obtain a more intuitive classification basis but also to find a breakthrough point to improve the efficiency of the research method in the next step and further carry out quality control on FFUSP, which may become an essential basis for the next stage of work.

Experimental data involved in this paper were obtained from the fetal ultrasound scanning video. The added nonstandard planes included images similar to the standard plane morphology and other morphological images, which increased the difficulty in identifying the standard plane and interfered with the classification experiment in this study. However, the experimental data used in this study, to a certain extent, represent the real-time images obtained by ultrasonic scanning. The composition of the experimental data in this study and the final experimental results indicates the possibility of real-time detection of FFUSP by this method, further reflecting this method's clinical potential.

It is concluded from the experiment that the accuracy of the proposed method for the classification of FFUSP is 94.67%, indicating that the texture feature fusion method can effectively predict and classify FFUSP, which provides an essential basis for clinical research on the automatic detection method of FFUSP. At the same time, there are still some shortcomings in this study. First, although the method used in this study performs well in the classification of FFUSP, it can only be used for rough classification. It cannot identify the specific anatomical structures in the standard planes. Second, the method used in this study still misclassifies some ultrasound images. Third, the experimental data in this study were all from pregnant women with a healthy fetus, and the recognition challenge of the standard plane was relatively small. Fourth, this study's experimental data volume is relatively small, so the proposed method cannot be compared with the deep learning model with the same data set.

In the next stage of our work, we will strive to overcome the above shortcomings. First of all, we will continue to establish a relatively standardized and sizeable ultrasound image database. We can compare and evaluate the performance of more different method models. Further, efforts are made to detect the standard plane's fundamental anatomical structures; we will use the similarity of plane prediction as the breakthrough point to identify and classify the images through the standard plane quality control. Fetal ultrasound images of more different pathological cases will be collected on experimental data. Besides, we will look for more effective ways to overcome the image differences caused by different ultrasonic instruments and different scanning techniques to pass the external examination as soon as possible.

## 5. Conclusion

To solve the problem that the traditional method of obtaining FFUSP is highly dependent on the doctor's seniority, energy, and other aspects, and save time and human resources; in this study, we used the fusion of LBP and HOG to extract the texture features of the image and SVM classifier for recognition and classification to achieve the rapid classification of FFUSP. We first collected a certain amount of data on standard and nonstandard planes of ultrasound of the fetal face. A senior sonographer strictly screened each ultrasound image. In this experiment, we have obtained the FFUSP recognition accuracy of 94.67%. To verify the stability of the experimental method, we performed experiments under different parameters. The results showed that the experimental method could still achieve excellent results under different parameters. The results obtained under 41 groups of parameters were stable. Besides, with the addition of nonstandard planes, which were very similar to the standard planes, the experimental results were still significant, which strongly verified this experimental method's clinical application potential. The proposal of the concept of prediction similarity lays the foundation for the next stage of work. The experimental results showed that this research method was a very effective method for the classification of FFUSP. It could further effectively solve the problem of the dependence of clinical acquisition of FFUSP on the doctor's seniority, energy, and other subjective factors.

## Figures and Tables

**Figure 1:** Image of FFUSP (a) OAP, where CL represents the crystalline lens and EB represents the eyeball; (b) MSP, where FB represents the frontal bone, NB represents the nasal bone, AN represents the apex nasi, and LJ represents the lower jawbone; (c) NCP, where AN represents the apex nasi, NC represents the nasal column, Nos represents the nostril, UL represents the upper lip, LL for lower lip, and MD for the mandible.

**Figure 2:** Process flow chart of this proposed method.

**Figure 3:** Image of N-SP. (a) Images similar to a standard plane shape. (b) Other forms of images.

**Figure 4:** Texture feature fusion schematic diagram.

**Figure 5:** Scatter plot of experimental results corresponding to different cell sizes.

**Figure 6:** Prediction and classification process of FFUSP.

**Table 1:** Data distribution in this lab set.

Class	Total	1	2	3	4	5
OAP	221	45	45	45	45	41
MSP	298	60	60	60	60	58
NCP	424	85	85	85	85	84
N-SP	350	70	70	70	70	70

**Table 2:** The results of this experimental method.

Method	Group	Precision (%)	Recall (%)	*F*1-score (%)	Accuracy (%)
The proposed (LH-SVM)	A	97.44	97.17	97.30	97.31
	B	93.74	93.10	93.38	94.23
	C	92.79	91.58	92.06	93.08
	D	92.02	91.71	91.85	92.69
	E	95.39	95.82	95.54	96.05
	AVG	94.27	93.88	94.08	94.67

**Table 3:** Comparative experimental results of different texture features and classifiers.

Methods		AVG-Pre (%)	AVG-Re (%)	AVG-*F*1 (%)	Accuracy (%)
Texture	Classifier				
LBP	SVM	93.45 (±2.61)	93.15 (±3.02)	93.25 (±2.86)	93.97 (±2.18)
HOG	SVM	89.87 (±2.26)	89.22 (±2.59)	89.45 (±2.51)	90.72 (±2.36)
LBP + HOG	SVM	94.27 (±3.17)	93.88 (±3.29)	94.03 (±3.27)	94.67 (±2.64)
LBP	KNN	88.96 (±2.90)	87.08 (±3.57)	87.66 (±3.47)	89.33 (±3.30)
HOG	KNN	89.31 (±3.57)	88.07 (±4.19)	88.42 (±4.05)	89.78 (±3.30)
LBP + HOG	KNN	90.32 (±0.88)	89.77 (±1.07)	89.95 (±0.75)	90.87 (±0.67)
LBP	NB	70.29 (±6.41)	70.65 (±6.07)	69.91 (±6.32)	72.68 (±6.14)
HOG	NB	73.73 (±3.55)	73.17 (±3.05)	73.25 (±3.33)	76.33 (±2.90)
LBP + HOG	NB	78.08 (±2.95)	77.34 (±3.64)	77.24 (±3.32)	79.81 (±2.88)

**Table 4:** Comparative experimental results of different (*P*, *R*) values of LBP (texture feature: LBP + HOG, classifier: SVM).

(*P*, *R*)	AVG-Pre (%)	AVG-Re (%)	AVG-*F*1 (%)	Accuracy (%)
(8, 1)	94.27 (±3.17)	93.88 (±3.29)	94.03 (±3.27)	94.67 (±2.64)
(16, 2)	93.72 (±2.52)	93.40 (±2.37)	93.52 (±2.44)	94.20 (±1.95)
(24, 3)	92.37 (±2.20)	91.98 (±1.68)	92.11 (±1.81)	93.04 (±1.58)
(8, 1) + (16, 2)	94.07 (±2.08)	93.60 (±2.17)	93.77 (±2.18)	94.52 (±1.63)
(8, 1) + (24, 3)	93.90 (±2.92)	93.64 (±2.77)	93.74 (±2.82)	94.44 (±2.52)
(16, 2) + (24, 3)	93.52 (±2.35)	93.23 (±1.98)	93.31 (±2.16)	94.13 (±1.64)

## Data Availability

The Fetal Facial Ultrasound Image data used to support the findings of this study were supplied by Quanzhou first hospital in Fujian, China, under license and so cannot be made freely available.
